# Metagenomic Analysis Reveals *Neisseria bacilliformis* Variation in the Early Childhood Caries Plaque Microbiome

This article has been retracted.

**DOI:** 10.1155/2021/2774772

**Published:** 2021-10-21

**Authors:** Xiaofen Xiao, Shandan He, Fei He, Xiaoyun Wu, Yuyan Zheng

**Affiliations:** ^1^Department of Stomatology, Shenzhen People's Hospital, Second Clinical Medical School of Jinan University, First Affiliated Hospital of Southern University of Science and Technology, Shenzhen, Guangdong 518020, China; ^2^Shenzhen People's Hospital, Second Clinical Medical School of Jinan University, First Affiliated Hospital of Southern University of Science and Technology, Shenzhen, Guangdong 518020, China

## Abstract

The progression of early childhood caries (ECC) is caused by microbial colonized in dental plaque. However, the association framework both from 16s genus down to high resolution metagenomic strain level and from composition to genome function analysis on caries lacks. 16S rRNA sequence revealed the composition of 3–6 years dental caries (ECC, *n* = 29), and severe dental caries (SECC, *n* = 36) children are significantly different from caries-free controls (CF, *n* = 31). Especially, genus *Neisseria* is enriched in caries (*P* < 0.05). Metagenomics sequence of 3 ECCs, 3 SECCs, and 3 CFs reveals *Neisseria bacilliformis* ATCC BAA-1200 in genus *Neisseria* is also significantly enriched in caries (*P* < 0.05). Then, we recovered high-quality metagenomic assembly genomes (MAG), named bin 86, which have 99% identity with *Neisseria bacilliformis* ATCC BAA-1200 genome. Function analysis of *Neisseria bacilliformis* ATCC BAA-1200 genome shows its metabolism power of sugar and adhesion, colonization, acid production, and acid tolerance ability, which suggested *Neisseria bacilliformis* ATCC BAA-1200 may serve as a biomarker for childhood caries.

## 1. Introduction

Dental caries is a classic bioﬁlm-induced disease that causes the decay of the mineralized tooth tissue [1]. Caries not only results in the dysfunction of the oral cavity system but also act as risk factors for a variety of diseases, such as digestive diseases, cardiovascular diseases, and kidney damage [2, 3]. Therefore, the prevention of dental caries is an emerging task in clinical research [4, 5]. Previous studies classified dental caries which predominantly affect preschool children as early childhood caries (ECC) [6]. The progression of ECC is painful and recurring, which may lead to severe tooth decay and result in the deconstruction of the total oral environment if left untreated. It is generally accepted that the bacteria in dental plaque forms the biofilm, which plays a crucial role in the initiation and progression of ECC [1, 7]. When children are overexposed to dietary sugars, the microbials residing in bioﬁlms are changed and prefer carbohydrates metabolization which produces acids destroying tooth tissues [1, 8]. However, our understanding of microbial diversity and composition in dental plaque derived from caries-free (CF) and ECC subjects is insufficient [9, 10].

With advances of next-generation sequencing technologies, recent studies have demonstrated that the composition of the bacterial community might play a crucial role in the progression of caries [1, 8]. Supragingival and saliva derived from the dental caries group have a more varied microbial community structure compared with the caries-free group [11]; a longitudinal study showed that the diversity of the bacterial community in saliva from different progressive stages is reduced [12]. However, Zhou et al. found a similar oral microbiota diversity in saliva among children with caries and without caries [13]. Therefore, our understanding of the association between bacterial diversity and dental caries is unclear and thus required a more in-depth exploration.

In this study, we profiled the composition of microbiota in dental plaque in children with and without dental caries and aimed to identify potential genus associated with caries using high-throughput sequencing of 16S rRNA genes and metagenomics. We characterized the diversity, composition, and PICRUSt function of dental plaque in CF, ECC, and SECC subjects. We also assembly and bin the metagenomics data into high-quality MAGs. Strain level MWAS was performed to figure out the specific genomes association with caries. The analysis of its genome function shows that it has a strong sugar metabolism and adhesion, colonization, acid production, and acid resistance, which is the basis for the formation of dental caries. We found that the strain *Neisseria bacilliformis* ATCC BAA-1200 is very important in childhood caries development. Our study provides insights into the vital role of oral microbiota in dental plaque of children with caries and benefit the prevention of ECC.

## 2. Materials and Methods

### 2.1. Ethical Approval of the Study Protocol

This study was independently reviewed and approved by the Ethical Committee of the Shenzhen People's Hospital and IRB of Shenzhen People's Hospital on April 6th, 2016 (#LL-KT-201682). All methods were performed in accordance with the relevant guidelines and regulations. Informed consent for participates was obtained from at least one parent prior to the oral health survey.

### 2.2. Study Design and Sample Collection

All participates were recruited from patients from Shenzhen people's hospital, Shenzhen, China, between June 2011 and June 2017. For each participate, we evaluated the oral health status through examining the teeth, oral mucosa, periodontal tissues, and reviewing medical histories, respectively. All participants aged from 3 to 6 years old and live in a homogeneous environment. The number of caries and missing fillings (DMFS) indicator, representing the presence of one or more decayed (noncavitated or cavitated lesions), missing (due to caries), or filled tooth surfaces in any primary tooth, was used to evaluate the degree of dental caries [14]. All participants in this study can be classified into three host groups based on their development of caries: CF group with no decayed (noncavitated or cavitated lesions), missing (due to caries), or filled tooth surfaces; ECC group with DMFS < 4 (age 3), DMFS < 5 (age 4), and DMFS < 6 and no decayed (noncavitated or cavitated lesions), missing (due to caries), or filled tooth surfaces in primary maxillary anterior teeth; and severe dental caries (SECC) group with DMFS in primary maxillary anterior teeth ≥ 1, or DMFS ≥ 4 (age 3), DMFS ≥ 5 (age 4), and DMFS ≥ 6 (age5). Dental plague samples from participates were extracted for downstream analysis.

### 2.3. DNA Extraction and High-Throughput Sequencing

Total DNA was extracted from dental plaque samples according to the protocol described in a previous study [15]. Briefly, the frozen dental plague samples were thawed on ice and then transferred into a clean bead-beating tube (Eppendorf, Germany). Freshly prepared lytic enzyme cocktail master mix was added and incubated at 37°C for 45 min. To lyse the microbiome of dental plaque samples, we added 750 mg cleaned and dry 0.1 mm diameter zirconia-silica beads to the above lysate mix and performed bead beating for 2 minutes at room temperature using a TissueLyser LT (Qiagen, Germany). The crude lysate (100 *µ*l) was transferred into a new tube, and DNA was isolated by QIAcube using DNeasy® blood and tissue mini kits. Amplicons spanning V3-V4 region of 16S rRNA gene sequence were amplified by the primers (forward: NNNNNNN-TGGAGAGTTTGATCCTGGCTCAG and reverse: NNNNNNN-TACCGCGGCTGCTGGCAC). Barcode sequences were then synthesized at the 5′ end of each pair of primers, which are unique for each sample. The barcoded 16S rRNA amplicons were sequenced using Illumina HiSeq 2500. For metagenomic sequencing, 0.5 *μ*g metagenomic DNA was sheared into fragments of ∼350 bp in length; then, a sequencing library was constructed according to a standard protocol provided by Illumina Inc. (San Diego, CA, USA). The libraries were then sequenced using illumine HiSeq 2500 with 2 × 250 bp paired-end (PE) sequencing.

### 2.4. DNA Extraction and Metagenomics Shotgun Sequencing

DNA extraction of the 10 dental samples was performed as above. Metagenomic sequencing was done on the HiSeq X Ten platform (150 bp of paired-end reads).

### 2.5. 16S rRNA Analysis

The adapter and low-quality bases were trimmed from 3′ to 5′ ends for the raw sequencing reads using Readfq (https://github.com/billzt/readfq). After trimming, reads shorter than 36 bp were discarded. Subsequently, the preprocessed reads were assembled to obtain raw 16S rRNA tags using FLASH [16]. To remove chimeric sequences, we aligned all tags to the GOLD database (https://gold.jgi.doe.gov/) using the UCHIME algorithm [17], and the chimeric tags were eliminated for further analysis. Then, operational taxonomic units (OUT) were constructed using UPARSE [18], and the filtered tags were mapped to the SILVA 16S rRNA database [19] to determine the tag counts for each OTU using the QIIME package (pick_closed_reference_otus.py) [20]. QIIME package was used to calculate the relative abundances of each OTU (summarize_taxa.py and summarize_taxa_through_plots.py). The NGS datasets have been deposited to sequence read archive in NCBI (accession id: SRP170994).

### 2.6. Metagenomic Assembly, Contig Binning, and Annotation

Raw reads were filtered as described above, and then, the filtered reads were used for downstream analyses. Briefly, the contaminated reads were removed if they were unambiguously aligned to the human reference genome (hg19); then, the remaining reads were subjected to a de novo assembly. Reconstruct bacterial and archaeal genomes from the dental microbiome exploits metagenomic single sample assembly and contig binning and applied metagenomic assembly MEGAHIT [21] to each sample separately. Each metagenomic assembly was then quality controlled for minimum length and were subjected to sample-specific contig binning metaWRAP (Uritskiy et al., 2018). We selected high-quality (HQ) genomes having completeness >70% and contamination <5% resulting in a total of 43 microbial genomes using CheckM (Parks et al., 2015) (version 1.0.7; lineage specific workflow). Genes were predicted from the assembled contigs using MetaGeneMark v2.8 [22] and then compared all predicted genes against the NR database using BLASTP. Only the best BLAST hits were retained, and functional annotation of these collected BLAST hits was subjected for the KEGG pathway [23] enrichment analysis. The functional comparison of predicted genes was carried out among CF, ECC, and SECC.

### 2.7. Statistical Analysis

To evaluate within-sample and between-sample diversity of microbial community in dental plague samples, we applied alpha_diversity.py (QIIME package) to calculate Shannon index for each sample and applied beta_diversity.py to calculate Bray–Curtis dissimilarity between samples [20]. Subsequently, we applied principal_coordinates.py (QIIME) to samples clustering through principal coordinate analysis. PERMANOVA statistical analysis was applied to sample categorization using compare_categories.py script in QIIME package [24]. For comparison analysis between groups, we first filtered out OTUs not present in at least 2 samples or lower than 1% abundance using ﬁlter_otus_from_otu_table.py in QIIME package. Then Kruskal–Wallis analysis was performed to evaluate the signiﬁcant changes in the relative abundance between sample groups using Metastats and group_signiﬁcance.py script in QIIME package [20, 25].

## 3. Result

### 3.1. The ECC or SECC Dental Bacterial Community Are Different Compared with CF

Recent studies have demonstrated that the changes of the bacterial composition might play a crucial role in the progression of caries [9, 10]; thus, it is necessary to investigate the bacterial diversity and composition in dental plaque derived from CF, ECC, and SECC. To this end, we applied 16 rRNA gene sequencing on 96 dental plague samples and obtained 5,964,124 high-quality tags with a mean read length of 418.7 bp. A total of 1,105 OTUs were generated through clustering analysis of all qualified sequences using 97% similarity cutoff. Then, we identified 1003, 992, and 1080 OTUs for CF, ECC, and SECC group, respectively; the three groups shared 82.5% of the total OTUs. The average coverage per sample was over 97%, suggesting that the identified 16S rRNA genes represent most bacterial taxa inhabiting the dental plague samples in the current study (Figure 1(d)).

We next explored the association between the dental microbiome structures and caries status. CF shows more intragroup diversity than the caries group (ECC or SECC) based on Bray–Curtis distance (Figure 1(b)). Intergroups accounted for the majority of variance for dental microbiomes based on unweight UniFrac distance. The bacterial composition between CF, ECC, and SECC was significantly different using Adonis or multiresponse permutation procedure (MRPP) analysis (Figure 1(c), Table S1). Both methods are commonly used to evaluate the difference of the diversity and structure of microbial community among groups. Although, the Shannon index was not impressive between groups (Figure 1(a)). Collectively, our analyses demonstrated that the bacterial community in dental caries (ECC and SECC) is different compared with the CF group, indicating that further exploration of the detailed map of the microbial community might explain the development of caries.

### 3.2. Multiple Genus including *Neisseria* Are Enriched in Childhood Caries

Previous research indicates a multispecies etiology for dental caries; the mutants *streptococci* (MS) are still recognized as major constituents of the most active dental caries lesions [24]. We found that *Streptococcus* is not significantly different among CF, ECC, and SECC (Figure S1). However, *Neisseria, Atopobium*, *Lactobacillus*, and *Veillonella* showed higher abundance in the caries group compared to the caries-free group (*P* < 0.05, Figure S1). *Neisseria*, *Veillonella*, and *Lactobacillus* were potential acid producers, which might be responsible for the decay of teeth. *Atopobium* [26] reported the strongest association with caries.

The linear regression model (PERMANOVA) [27] was carried out to investigate the correlation between genus marker and medical index. We found that caries-enriched genera *Veillonella* and *Lactobacillus* show a significant correlation with DMFS index, despite gender and age (Figure S2). *Bifidobacterium*, *Scardovia*, and *Selenomonas* also significantly correlate with DMFS. *Bifidobacterium* [28] are reported enriched in caries samples. Our data again indicated that dental microbes play an important role in the progression of caries.

### 3.3. Elevated Carbohydrate Metabolisms in Caries-Related Microbiome

Recent studies have demonstrated that the changes of microbial communities can disrupt the host microbial homeostasis to cause caries [1, 8], but how the changes of microbial communities affect the microbial homeostasis in dental plaque requires further investigation. To this end, we predicted the function profile of 16 s data using PICRUSt. We investigated the functions of oral microbiota in dental plague of caries. KEGG enrichment analysis showed that the carbohydrate metabolism (propanoate metabolism and glyoxylate and dicarboxylate metabolisms) and metabolism of other amino acids (selenocompound metabolism) were enriched in ECC dental microbiomes compared with CF, while cell cycle, *Caulobacter*, and bacterial secretion system were depleted in ECC (*q* value <0.1, Table S2). These support the hypothesis that sugar eating habit will increase strong carbohydrate metabolisms microbes.

Strain-level structure and function of the dental microbiome reveal *Neisseria bacilliformis* ATCC BAA-1200 associated with caries.

Metagenomics sequence enables us to find crucial differences present at the strain level only. Strains are known that typical intraspecies genomic variability can result in wide range of phenotypic diversity, including virulence, substrate utilization, antibiotic production, or susceptibility [29–31]. As the result, we assembled and combined 43 high-quality metagenomics assembly genomes (MAG) (completeness >70% and contamination <5%) from 3 ECC, 4 SECC, and 3 CF individuals (Table S3). 3 MAGs were from caries enriched genera *Neisseria*, *Veillonellaceae,* and *Lactobacillaceae* as described above. 2 MAGs were from previous report caries-related *Streptococcus*. 1 pathogen MAG was from *Capnocytophaga*. Unexpectedly, 10 MAGs were from *Actinobacteria,* which were potential lactic acid producers. 9 MAGs were from Prevotellaceae (Figures 2(a) and S3).

We next explored these MAGs' association with caries status in strain levels. *Neisseria bacilliformis* ATCC BAA-1200 (MAG: bin 86) were significantly enriched in caries groups compared with caries free (*P* < 0.05, Figure 2(b)), which validated the 16s genus biomarkers. *Neisseria bacilliformis* ATCC BAA-1200 (bin 86) were also positive correlated with DMFS index (Figure S3). Using NCBI BLAST, MAG (bin 86, 91% completeness, 1.8% contamination, 60.2% GC, N50 18117b, size 2105996b) hits 99% identify with *Neisseria* bacilliformis ATCC BAA-1200 genome. Besides, *Streptococcus sobrinus* (bin 3), *Bifidobacteriaceae* (bin 59), and 3 MAGs belonging to *Actinobacteria* (bin 33, bin 63, and bin 40) were also enriched in caries groups, which were not found in 16s genus biomarkers, and may suggest the strain variance in these genera. *Actinobacteria* are reported to produce lactic acid and strong adhesive properties.

Next, we explored their function association with caries from genome view. Dental caries is a biofilm infectious disease, and virulence factors are closely related to biofilms, such as surface proteins P1 (PAC) and glucosyltransferases (GTFs). They are associated with adhesion colonization and related to acid production, lactate dehydrogenase (LDH), and acid-related proton-translocating ATPase [32]. We found *Neisseria bacilliformis* ATCC BAA-1200 genome (MAG: bin 86) were positive correlated with the glucose-related metabolism pathway (glycosaminoglycan biosynthesis–keratin sulfate, other glycan degradation, N-glycan biosynthesis, various types of N-glycan biosynthesis, pentose phosphate pathway, stilbenoid diarylheptanoid, and gingerol biosynthesis), which may indicate that *Neisseria bacilliformis* ATCC BAA-1200 (MAG: bin 86) has the acid production capacity by fermented sugar (Figures 3(a) and S4). Besides other caries enriched MAGs such as *Streptococcus sobrinus* (bin 3), Bifidobacteriaceae (bin 59) are also positively correlated with the glucose-related metabolism pathway. We also count the occurrence of virulence factor genes in adhesion, colonization, acid production, and acid tolerance in caries enriched MAGs (Figure 3(b)). We found *Neisseria* sp. *KEM232* (MAG: bin 86) contained highest number of VF genes among other MAGS. Acid durance and adhesion are the premise of continuous acid production and foundation of caries. In summary, our result showed that the disturbance of metabolism maybe an important factor for microbial colonization and biofilm formation in caries subjects, which is useful for further investigation of the progression of ECC.

## 4. Discussion

In this study, we had assessed the composition of microbiota community of dental plague, which is very important for the development of caries in children. We observed a significant difference of bacterial composition among CF, ECC, and SECC children through a beta-diversity analysis. We identified genera that are specifically associated with SECC. Genus *Neisseria* are significantly enriched in caries, besides other genera *Atopobium*, *Lactobacillus,* and *Veillonella* are also enriched in dental plague, which confirmed previous multiple species results that lead to the progression of caries. Furthermore, genera *Veillonella, Lactobacillus*, and *Bifidobacterium* were positively correlated with DMFS index. PICRUSt analysis shows that these genera have high carbohydrate metabolisms ability, which may promote the acid producing and forming caries. These data therefore characterize how caries are associated with microbial species in dental plague of ECC and SECC. Our hope is that the species with high abundance in ECC and SECC will serve as candidates in future studies for prophylactic targets that can potentially prevent the progression of ECC.

In addition, we preformed metagenomic sequencing of the dental plague sample. We identified 43 high-quality MAGs. Although the small sample size of the metagenomics samples limited the confidence of the results, strain level analysis will provide us some hints, in which genomes are the center species responses for caries. Specific genomes belonging to the above genus are also significantly enriched in caries children. Among them, function analysis of *Neisseria bacilliformis* ATCC BAA-1200 (MAG: bin 86) genome shows metabolism power of sugar and adhesion, colonization, acid production, and acid tolerance ability. These genes help in hemostasis of microbial colonization and the formation of biofilm in the dental plaque of caries subjects.

In summary, our analysis of the microbiota community in the dental plague sample should be useful for the prevention of ECC, which may help in the improvement of child healthcare.

## Figures and Tables

**Figure 1:** Diversity analysis of plaque samples from CF (*n* = 31), ECC (*n* = 29), and SECC (*n* = 26). (a) Comparison of the Shannon index among CF, ECC, and SECC. (b) Intragroup diversity based on Bray–Curtis distance. (c) PCOA of unweight UniFrac distance. (d) The distribution of genera in CF, ECC, and SECC. Bar plot shows the fraction of different genera in CF, ECC, and SECC.

**Figure 2:** Metagenomics-wise strain level association with caries. (a) Quality control of metagenomics assembly genomes (MAG). (b) Strains association with caries. The box depicts the interquartile range (IQR) between the first and third quartiles (25th and 75th percentiles, respectively) and the line inside denotes the median, whereas the points represent the abundance of sample.

**Figure 3:** Function analysis of MAGs. (a) Heatmap of spearman correlation between function profile and strain abundance profile. (b) Heatmap of gene numbers of genomes annotation to adhesion, colonization, acid production, and acid tolerance.

## Data Availability

The data used to support the findings of this study are available from the corresponding author upon request.

## Supplementary Materials

Supplementary Materials Figure S1. Genus biomarkers for caries. The box depicts the interquartile range (IQR) between the first and third quartiles (25th and 75th percentiles, respectively) and the line inside denotes the median, whereas the points represent the abundance of sample. Figure S2. Association between genus biomarkers and decayed, missing, and filled surface (DMFS) index. Heatmap of the spearman correlation between genus and DMFS, age, and gender. BH adjusted *P* value is denoted: ^+^*q* value <0.1; ^*∗*^*q* value <0.05; ^*∗∗*^*q* value<0.01. Figure S3. MAGs population distribution. Heatmap of relative abundance of MAGs. Figure S4. Association between pathway and caries. Heatmap of the spearman correlation between pathway and caries. The Wilcoxon test was used to compare groups. BH adjusted *P* value is denoted: ^+^*q* value<0.1; ^*∗*^*q* value<0.05; ^*∗∗*^*q* value<0.01. Supplementary Table S1. ANOSIM analysis of the difference among CF, ECC, and SECC. Supplementary Table S2. Significant pathway between CF, ECC, and SECC groups. Supplementary Table S3. Basic statistics of samples for metagenome sequencing. .
